# Application of High-Quality Nursing Intervention Based on Humanistic Care Combined with the Project Teaching Method in Patients with Acute Leukemia Undergoing Chemotherapy

**DOI:** 10.1155/2022/2972037

**Published:** 2022-02-09

**Authors:** Zhiyan Wang

**Affiliations:** Department of Hematology Oncology, Tianjin Fifth Central Hospital, Tianjin 300450, China

## Abstract

Chemotherapy, the main treatment method of AL, can produce varying degrees of toxic and side effects on patients while killing tumor cells, resulting in decreased immune function of patients. We aim to explore the application effect of high-quality nursing intervention based on humanistic care combined with the project teaching method on patients with acute leukemia (AL) undergoing chemotherapy and its effect on their psychological state and satisfaction. 114 AL patients undergoing chemotherapy in the Department of Hematology of our hospital from July 2018 to July 2020 were chosen as the research objects and equally randomized into the experimental group (EG) and control group (CG). CG received routine nursing during chemotherapy, while EG received high-quality nursing intervention based on humanistic care combined with the project teaching method. Hospital Anxiety and Depression Scale (HAD) was adopted to evaluate the psychological state of patients in both groups after intervention, and the self-made nursing satisfaction questionnaire in our hospital was applied to evaluate the clinical nursing satisfaction. The HAD-A and HAD-D scores in the CG (*P* < 0.001) were significantly higher than the HAD-A and HAD-D scores in the EG after intervention. The scores of various coping styles in the EG after intervention were better than those in the CG (*P* < 0.05). Compared with the CG, the total nursing satisfaction after intervention was remarkably higher in the EG (*P* < 0.001), while the total incidence of adverse reactions during intervention was notably lower (*P* < 0.05). High-quality nursing intervention based on humanistic care combined with the project teaching method for AL patients undergoing chemotherapy can effectively relieve negative emotions, improve clinical nursing satisfaction, and reduce adverse reactions during chemotherapy.

## 1. Introduction

Acute leukemia (AL), a common malignant tumor of hematopoietic stem cells, often presents with symptoms such as bleeding, anemia, infiltration, and infection [1]. We can clinically split AL into two parts according to the cell types involved: acute lymphoblastic leukemia (ALL) and acute myeloid leukemia (AML). The primary symptoms of AL included persistent high fever or repeated infection with enlargement of the spleen, liver, and lymph nodes to varying degrees, resulting in only a few months of survival time in most patients without treatment. Chemotherapy is a common treatment method for AL to inhibit tumor growth in patients [2]. A clinical study [3] has shown that although the condition in 65% of patients can be effectively alleviated after the first chemotherapy and 20% of the patients can live for more than five years, there are also a high recurrence rate and incidence of adverse reactions, affecting the treatment compliance and quality of life of patients and leading to depression. Since negative emotions can make the psychological state of patients more vulnerable, strengthening the nursing intervention for such patients during chemotherapy is convincing to reduce negative emotions and increase the therapeutic effect [4–6]. High-quality nursing intervention based on humanistic care pays attention to the changes of patients' physical and mental feelings, enables them to feel the care from medical staff through various nursing means, and improves their nursing satisfaction, which has been confirmed in patients with radical mastectomy [7]. The project teaching method is centered on team learning, takes course projects as the main line, takes task goals as the mission, and emphasizes the ability, quality, and professional knowledge of medical staff. It can effectively cultivate nurses' sense of teamwork and innovation and improve nursing satisfaction, which has been proved in advanced cancer [8]. Modern society attaches great importance to teamwork and innovation and requires all team members to cooperate actively with each other to form the highest synergy effect. Some scholars [9, 10] pointed out in their studies that many students expressed that the project teaching method, especially the thinking mode of highlighting team characteristics by naming clinical departments, reduced the strangeness and fear of clinical practice and made them quickly adapt to clinical nursing. Be founded on this, this study proposes to investigate the application effect of high-quality nursing intervention based on humanistic care combined with the project teaching method on AL patients undergoing chemotherapy and its effect on their psychological state and satisfaction.

## 2. Materials and Methods

### 2.1. Data Collection

In this prospective randomized controlled clinical study, we selected 114 AL patients undergoing chemotherapy in the Department of Hematology of our hospital from July 2018 to July 2020. The inclusion criteria were as follows: (1) the patients satisfied the powerful diagnostic criteria of AL in *Leukemia Diagnostics* [11], confirmed by bone marrow puncture; (2) the patients were no more than 65 years old; (3) the anticipated survival time of the patients was more than 3 months; (4) the patients did not receive antitumor drugs, biological immunotherapy, or other drug treatments before admission; (5) the patients received national uniform regimens of chemotherapy, with methotrexate as the main chemotherapy drug; and (6) the study conformed with the hospital ethics institutional mechanisms, and the patients knew and approved informed consent. The exclusion criteria were as follows: (1) the patients with allergy to chemotherapy drugs; (2) the patients complicated with liver, kidney, cardiopulmonary, and brain dysfunction; (3) the patients with mental and other cognitive dysfunctions; and (4) the patients complicated with other malignant tumors.

### 2.2. Methods

The patients in the CG received routine nursing during treatment. After admission, they were informed of the hospital conditions (hospital environment and hospital rules and regulations), the specific process, adverse reactions, and precautions of chemotherapy in detail. The health education paths for patients with chemotherapy were developed by the medical staff of the department, including disease cognition, medication management, diet management, and psychological nursing, and education was carried out through distribution of health promotion manuals and centralized or individual oral education. The patients also received monitoring of the vital signs, basic drug nursing and life nursing, and appropriate treatment of complications [12–14].

The patients in the EG received high-quality nursing intervention based on humanistic care combined with the project teaching method. The specific steps of high-quality nursing based on humanistic care were as follows. (1) The actual needs of patients were analyzed to master their specific psychological status, mental state, and their own cognition of the disease. Medical staff communicated with patients (1 time/day and 15 min each time) to understand their real thoughts and needs and encourage them to bravely express their feelings. The staff also provided timely nursing for patients and their families, improved their quality of life during chemotherapy, reduced the side effects of chemotherapy, respected their original lifestyles as much as possible, and arranged them to do what they could do according to their condition. The staff should have enough patience to understand the patients' emotions. (2) Targeted programs should be adopted according to different psychological emotions of patients to timely solve their psychological problems, eliminate adverse emotions, and reduce their fear of chemotherapy. Meanwhile, the staff should also carry out death education for patients to eliminate their anxiety and fear when facing death, which could also help their families to ease their grief. (3) The pain of patients during chemotherapy was minimized, and analgesic treatment should be carried out for patients who could not tolerate the pain. If the pain of patients was not alleviated, other analgesic schemes could be adopted, or other analgesic methods could be applied jointly, such as slow breathing and distraction. Necessary care and concern were given to patients. In addition to drug treatment, appropriate comfort should be provided when the pain occurred during chemotherapy, which reflected humanistic care. Besides, targeted nursing measures should be taken to reduce the physical pain of patients and soothe their bad emotions. (4) The family members were instructed to make food with high vitamin and protein contents for patients. Food should be easy to digest and not be too greasy, with more fresh fruits and vegetables. The wards were kept quiet, clean, and comfortable with appropriate temperature and humidity. The patients were advised to keep adequate sleep every day and walk properly in the wards if circumstances permitted to relieve the gastrointestinal discomfort caused by chemotherapy. (5) The patients with adverse reactions after chemotherapy should be actively intervened by strengthening perianal, perineal, and oral nursing. For example, the patients were advised to brush their teeth before and after eating and before sleeping, rinse the mouth with salt water, and maintain normal defecation to prevent constipation. Before chemotherapy, they orally took omeprazole to reduce the damage to gastric mucosa. The number of vomiting and the nature of vomit were carefully recorded, and the changes in skin color were observed [15–17].

Project teaching method was implemented as follows. (1) According to the clinical situation of typical cases, clinical teaching projects were formulated. The nurse with more than 6 years of experience in the department acted as the team leader, and other team members were nursing staff in the department to dynamically observe the information of patients in each ward. In this study, taking AL patients who underwent chemotherapy as an example, since the project was to develop the nursing plans for such patients, the team leader should consider the following aspects in the selection of cases. (a) The typicality of the disease: since the focus of the training was to cultivate the clear clinical thinking ability of the nursing staff, the cases should not be too complex. (b) The stability of the disease: the treatment pain of the patients should not be increased due to the project teaching. (c) Oral informed consent of patients and their families: the project teaching method started from the project selection, and the team leader should actively invite the team members to participate in the teaching project selection. (2) Teaching projects: they included teaching content, exploring projects, discussing problems, teaching operation, practical operation of team members, primary nurses, and expansion of new knowledge and new technology. (3) Division of teaching projects: guided by the team leader, each member of the group played a corresponding role and completed the task in the teaching projects. Every two nurses could undertake a task for supplement and comparison and carry out training on nurse-patient communication skills and humanistic care. (4) The nursing staff followed the doctors to make ward rounds and collect various clinical information of patients. If there were any doubts, they should timely consult the team leader and formulate nursing measures. The nursing measures should be matched with the problems one by one, which should be symptomatic, effective, economical, and operable, until the nursing plans were improved [18].

### 2.3. Evaluation Indexes

The anxiety and depression of patients before and after intervention were evaluated by referring to the Hospital Anxiety and Depression Scale (HAD) score [19]. The scale was divided into the HAD-A (for anxiety) score and HAD-D (for depression) score, with a sum of 15 points for each. The higher the score is, the more serious the negative emotions are.

The medical coping mode questionnaire (MCMQ) [20] was adopted to evaluate the coping styles of patients before and after intervention, including 20 items in three dimensions of avoidance, surrender, and facing and each scoring 4 points. The higher the score, the stronger the corresponding dimension.

The self-made nursing satisfaction questionnaire in our hospital was used to evaluate the satisfaction of both groups with clinical nursing. The full score of the questionnaire was 100 points, and a score of 80–100 points showed the patients were fully satisfied, with 60–79 as satisfied and 0–59 as dissatisfied. Total percentage of satisfaction = (fully satisfied cases + satisfied cases)/sum of cases × 100%.

### 2.4. Statistical Methods

The whole collected data were statistically analyzed and operated by SPSS 21.0 software and graphed by GraphPad Prism 7 (GraphPad Software, San Diego, USA). Enumeration data were tested by *X*^2^ and represented as *N* (%), while measurement data were tested by the *t*-test and expressed as ($\bar{x}\pm s$). The differences were statistically significant at *P* < 0.05.

## 3. Results

### 3.1. Comparison of Baseline Data

There are no obvious dissimilarities in sex ratio, average course of the disease, severity of the disease, disease types, marital status, residence, and education between the two groups (*P* > 0.05; Table 1).

### 3.2. Comparison of HAD Scores before and after Intervention

The HAD-A and HAD-D scores in the EG were obviously different before and after intervention (*P* < 0.001), and the scores in the EG after intervention were significantly lower than the CG (*P* < 0.001; Figure 1).

### 3.3. Comparison of Coping Style Scores before and after Intervention

The scores of various coping styles in the EG after intervention were better than those in the CG (*P* < 0.05; Table 2).

### 3.4. Comparison of Clinical Satisfaction

Compared with the CG, the total satisfaction after intervention was remarkably higher in the EG (*P* < 0.001; Table 3).

### 3.5. Comparison of the Occurrence of Adverse Reactions during Chemotherapy

The entire incidence of unfavorable reactions in the EG during intervention was remarkably lower than in the CG (*P* < 0.05; Table 4).

## 4. Discussion

AL will increase the psychological burden of patients and inevitably bring psychological and physiological stress responses to them. The pain caused by chemotherapy will increase the degree of stress response and affect the treatment compliance of patients [21]. AL patients should receive chemotherapy as early as possible to inhibit tumor growth, delay disease progression, and improve survival rate. However, some scholars [22] have found that chemotherapy drugs have both positive and negative effects, which can induce apoptosis of tumor cells, increase the release of 5-hydroxytryptamine in enterochromaffin cells, and activate 5-hydroxytryptamine receptors in the central nervous system, leading to a series of gastrointestinal adverse reactions. Studies [23, 24] have confirmed the high 5-hydroxytryptamine level in blood of patients with mental depression, which demonstrates that reducing the 5-hydroxytryptamine level can be achieved by improving patients' adverse emotions, thereby reducing gastrointestinal adverse reactions. Therefore, effective nursing intervention measures can increase the adverse emotions of AL patients, decrease the toxic and side effects of chemotherapy, and improve the therapeutic effect.

In this study, high-quality nursing intervention based on humanistic care combined with the project teaching method was implemented for patients in the EG. After intervention, the anxiety and depression of patients were remarkably improved because the high-quality nursing intervention based on humanistic care can provide high-quality clinical nursing support for AL patients undergoing chemotherapy, strictly implement the core idea of patient-centered nursing, provide emotional support for them, improve their psychological, spiritual, and physiological comfort, and enhance the nursing quality. In addition, in terms of coping styles, the symptomatic nursing for patients enabled them to face death directly and improve the courage and confidence of treatment. Therefore, the scores of various coping styles in the EG after intervention were better than those in the CG (*P* < 0.05), which was consistent with the study of Yang et al. [25]. The project teaching method simulates the clinical nursing team management so that nurses can quickly adapt to work. In this study, the total satisfaction after intervention was remarkably higher in the EG than in the CG (*P* < 0.05), suggesting that the combined intervention can help patients improve nursing satisfaction while eliminating their adverse emotions so that they can better cooperate with the treatment.

## 5. Conclusion

In conclusion, high-quality nursing intervention based on humanistic care combined with the project teaching method for AL patients undergoing chemotherapy can effectively relieve negative emotions and promote the development of positive coping styles, with high nursing satisfaction, which is worth applying and promoting. However, this study also has several limitations, such as the small sample size and lack of long-term follow-up observation of patients. Thus, we should expand the sample size with longer follow-up time to make the research results more objective.

## Figures and Tables

**Figure 1:** Comparison of HAD scores before and after intervention ($\bar{x}\pm s$). (a) Comparison of HAD-A scores before and after intervention. The abscissa described before and after intervention, and the ordinate described the HAD-A score (points). The HAD-A scores of the EG before and after treatment were 7.21 ± 1.83 and 4.62 ± 0.81, while those of the CG were 7.24 ± 1.92 and 6.94 ± 1.32. ^*∗*^A notable difference in the HAD-A scores of the EG before and after intervention (*t* = 9.771, *P* < 0.001); ^*∗∗*^a significant dissimilarity in the HAD-A scores after intervention (*t* = 7.827, *P* < 0.001). (b) Comparison of HAD-D scores before and after intervention. The abscissa described before and after intervention, and the ordinate described the HAD-D score (points). The HAD-D scores of the EG were 7.28 ± 1.83 before treatment and 5.13 ± 1.45 after treatment, while those of the CG were 7.23 ± 1.54 and 6.92 ± 1.36. ^*∗*^A notable difference in the HAD-D scores of the EG before and after intervention (*t* = 6.952, *P* < 0.001); ^*∗∗*^a notable difference in the HAD-D scores after intervention (*t* = 6.798, *P* < 0.001).

**Table 1:** Comparison of baseline data (*n* (%)).

Items	EG (*n* = 57)	CG (*n* = 57)	*X* ^2^/*t*	*P*
Gender			0.141	0.708
Male	31 (54.39%)	29 (50.88%)		
Female	26 (45.61%)	28 (49.12%)		
Average age ($\bar{x}\pm s$, years old)	32.67 ± 2.76	32.83 ± 2.69	0.313	0.755
BMI (kg/m^2^)	21.46 ± 1.64	21.48 ± 1.59	0.066	0.947
Average course of the disease (weeks)	3.46 ± 0.35	3.51 ± 0.28	0.842	0.402
Severity of the disease				
High risk	31 (54.39%)	29 (50.88%)	0.141	0.708
Medium risk	22 (38.60%)	23 (40.35%)	0.037	0.848
Low risk	4 (7.02%)	5 (8.77%)	0.121	0.728
Disease types			0.035	0.851
AML	27 (47.37%)	28 (49.12%)		
ALL	30 (52.63%)	29 (50.88%)		
Marital status				
Unmarried	9 (15.79%)	11 (19.30%)	0.243	0.622
Married	43 (75.44%)	42 (73.68%)	0.046	0.830
Divorced	5 (8.77%)	4 (7.02%)	0.121	0.728
Residence			0.141	0.708
Urban area	26 (45.61%)	28 (49.12%)		
Rural area	31 (54.39%)	29 (50.88%)		
Education				
College and above	17 (29.82%)	19 (33.33%)	0.162	0.687
High school	33 (57.89%)	29 (50.88%)	0.566	0.452
Middle school and below	7 (12.28%)	9 (15.79%)	0.291	0.590

**Table 2:** Comparison of coping style scores before and after intervention ($\bar{x}\pm s$, points).

Group	Facing		Surrender		Avoidance	
	Before intervention	After intervention	Before intervention	After intervention	Before intervention	After intervention
EG (*n* = 57)	14.28 ± 3.18	22.16 ± 3.14	21.16 ± 2.18	14.28 ± 1.87	13.28 ± 2.23	7.59 ± 1.58
CG (*n* = 57)	14.31 ± 3.09	16.25 ± 2.78	21.19 ± 2.11	17.26 ± 2.18	13.32 ± 2.35	11.02 ± 1.47
*t*	0.051	10.639	0.075	7.833	0.093	11.100
*P*	0.959	<0.001	0.941	<0.001	0.926	<0.001

**Table 3:** Comparison of clinical satisfaction (*n* (%)).

Group	*n*	Fully satisfied	Satisfied	Dissatisfied	Total satisfaction
EG	57	19 (33.33%)	36 (63.16%)	2 (3.51%)	96.49% (55/57)
CG	57	20 (35.09%)	28 (49.12%)	9 (15.79%)	84.21% (48/57)
*X* ^2^					4.930
*P*					<0.05

**Table 4:** Comparison of the occurrence of unfavorable reactions during chemotherapy (*n* (%)).

Group	*n*	Myelosuppression	Gastrointestinal discomfort	Cardiotoxicity	Respiratory tract infection	Total incidence
EG	57	1 (1.75)	2 (3.51)	0 (0.00)	1 (1.75)	7.02% (4/57)
CG	57	3 (5.26)	4 (7.02)	3 (5.26)	3 (5.26)	22.81% (13/57)
*X* ^2^						5.600
*P*						0.018

## Data Availability

The datasets used and/or analyzed during the current study are available upon request to the author.
